The article "The Identification of Chinese Herbal Medicine Combination Association Rule Analysis Based on an Improved Apriori Algorithm in Treating Patients with COVID-19 Disease" was published in 2022. Journal: J Healthc Eng.

# The Identification of Chinese Herbal Medicine Combination Association Rule Analysis Based on an Improved Apriori Algorithm in Treating Patients with COVID-19 Disease

**DOI:** 10.1155/2022/6337082

**Published:** 2022-08-31

**Authors:** Yanyan Zheng, Ying Chen

**Affiliations:** Department of Computer Science, Taizhou University, Taizhou 318000, China

## Abstract

In this work, an improved Apriori algorithm is proposed. The main goal is to improve the processing efficiency of the algorithm, and the idea and process of the Apriori algorithm are optimized. The proposed method is compared with the classical association rule algorithm to verify its effectiveness. Traditional Chinese medicine plays a certain role in the prevention and treatment of COVID-19. In order to deeply mine the association rules between Chinese herbal medicines for the prevention and treatment of COVID-19, this improved Apriori algorithm is applied from the retrieved published scientific literature and the guidelines for the prevention and treatment of COVID-19 published all over China. Based on the representation of traditional Chinese medicine data in binary form, the potential core traditional Chinese medicine combinations in the treatment of COVID-19 are identified. The results of association rules of Chinese herbal medicine data obtained from the real database provide an important reference for the analysis of COVID-19 combined treatment of Chinese herbal medicine.

## 1. Introduction

In recent years, under the background of the re-recognition of the value of Chinese traditional medicine [1] and the gradual maturity of data mining technology, in order to promote the further development of traditional Chinese medicine and realize the modernization of traditional Chinese medicine, the research in the field of traditional Chinese medicine data mining is gradually active. Researchers have gradually realized the combination of data mining, machine learning, artificial intelligence, and other technologies in the research field of traditional Chinese medicine. They hope to discover the hidden principles and laws through mining, analysis, induction, and summary of a large number of clinical experience data accumulated by traditional Chinese medicine workers for thousands of years.

Since December 2019, many pneumonia cases of unknown origin have been found in many countries and regions around the world. On February 11, 2020, the disease caused by the new coronavirus was officially named coronavirus disease-19, referred to as COVID-19 [2]. The pandemic has wrought serious negative effects on the global economy and society.

As a well-practiced therapeutic modality, traditional Chinese herbal medicines play a complementary role in alleviating the symptoms of certain diseases and improving the health-related quality of life among COVID-19 patients [3]. It has been widely accepted that the choice and combination of Chinese herbal medicines are vital for successful Chinese drug treatment [4]. The principles for choosing and combining Chinese herbal medicines are based on the Biaoben theory [5] and Meridian theory [6] in ancient Chinese therapy.

The Apriori algorithm is a type of association rule mining algorithm, and it proceeds by identifying the frequent individual itemsets in the database [7]. The Apriori algorithm is often used to analyze the combination of prescriptions and acupuncture points in the treatment of diseases by traditional Chinese medicine.

The Apriori algorithm is widely used in many fields, for example, to explore the main influencing factors and the interaction of factors in dangerous driving conditions of urban traffic [8], in the causal analysis of bridge deterioration [9], the employment trend analysis of college graduates [10], analysis of fault items in power optical transmission network [11], finding frequent patterns in live transportation data [10], and in the mining of association rules applied in traditional Chinese medicine. For example, prescription analysis for the treatment of impotence [12], optic atrophy [9], and so on [13–17]. The Apriori algorithm is often used to analyze the combination of prescriptions and acupuncture points in the treatment of diseases by traditional Chinese medicine.  Table 1 shows the differences between relevant studies and this study.

Starting from the comprehensive consideration of the redundancy of traditional Chinese herbal medicines treatment medicine data and the difficulty of rule mining, this article optimizes the idea and process of the Apriori algorithm with the goal of improving the processing efficiency of the algorithm and deeply mining the association rules between Chinese herbal medicines, and puts forward an improved Apriori algorithm. The improved algorithm is simulated and compared with the classical Apriori algorithm to verify its effectiveness. The calculated association rule results of Chinese herbal medicine point data provide an important reference basis for the analysis of Chinese herbal medicine combination in the treatment of COVID-19.

Section 1 introduces some background and presents some related work.  Section 2 gives some concepts of association rules.  Section 3 describes the improved Apriori algorithm.  Section 4 demonstrates the case study and result analysis. Finally, Section 5 concludes the article.

## 2. Problem Description and Basic Theory of Association Rules

### 2.1. Association Rules

Association rule mining is a basic data mining method used to mine interesting associations or correlations between itemsets from large-scale data sets. It is very helpful for data classification, clustering, and other data mining tasks.

The formal description of association rules is as follows [10–12]:

Dataset *D* is a collection of all things in the database. Each attribute of each record in the dataset is called an item, and the collection of attributes is called an itemset. Each nonempty record is called a transaction *T*.

Let *X* and *Y* be the two itemsets contained in transaction *T*, that is, *X* and *Y* are both proper subsets of *T*. If *X* is a nonempty subset, *Y* is also a nonempty subset, and the intersection of *X* and *Y* is an empty set, then *X*- > *Y* constitutes an association rule in the thing set *T*.

#### 2.1.1. Support

This is to say that an association rule is an expression in the form of *X* - > *Y*, where *X* is called the preceding term and *Y* is called the following term. The probability that both *X* and *Y* are contained in the itemset is called the support of *X* - > *Y*, denoted support (*X* - > *Y*) = *P* (*X* - > *Y*).

#### 2.1.2. Confidence

Under the condition that the prerequisite *X* of the association rule occurs, the probability that the association result *Y* occurs, that is, the probability that the itemset containing *X* contains *Y* at the same time, is called the confidence level of association rule *X* - > *Y*, denoted as confidence (*X*- > *Y*).

#### 2.1.3. Lift

The ratio of the possibility of including *Y* under the condition of *X* and the possibility of having *Y* in the itemset without this condition is called the lift of the association rule, denoted as Lift (*X*- > *Y*) = *P*(*Y* |*X*)/*P* (*Y*) = conference (*X* - > *Y*)/P (*Y*).

Association rule mining can usually be regarded as two basic processes: ① find all frequent itemsets from the transaction set, that is, find all itemsets whose support is greater than the given minimum support threshold; ② use the frequent itemsets found in the first step to generate all association rules, and the association rules that meet the minimum confidence are the strong association rules to be mined.

### 2.2. Apriori Algorithm

The algorithm uses a layer-by-layer search iterative method to find the largest *k*-term frequent set. First, the database is traversed and searched to get the candidate 1 itemset and its support. If its support is lower than the minimum support, it is pruned to get the frequent *1* itemset. Then, the obtained frequent *1* itemsets are connected to obtain the candidate *2* itemsets and their support, and so on. This is iterated until the frequent *K* *+* 1 itemsets cannot be obtained, and the corresponding frequent *K* itemset is the output result [9, 13, 14].

The Apriori algorithm's a priori property is that the subset of all frequent itemsets must be frequent itemsets. According to the properties, a corollary is obtained that the superset of infrequent itemsets must be infrequent [15, 16]. Using this property and inference, we can mine all levels of frequent itemsets that meet the threshold of support and credibility.

Apriori algorithm is widely used in many fields, [17], [18], [19] as mentioned above, and the mining of association rules applied in traditional Chinese medicine are basically Apriori algorithms. For example, prescription analysis for the treatment of peptic ulcers [20], leukaemia [21] and so on.

## 3. The Improved Apriori Algorithm

### 3.1. The Idea of the Improved Apriori Algorithm

Generally, the ways to improve the process of mining frequent itemsets include reducing the generation of candidate itemsets and reducing the number of transaction records to be compared when obtaining itemset support. The improved ideas are as follows.

1. Strong association rules are established, unrelated single transaction items are deleted, some association relationship between items is found, and their association is mined. In the process of generating frequent items, the Apriori algorithm needs to scan the huge transaction dataset many times and delete irrelevant transaction items, so as to reduce the dataset to a certain extent and improve the operation efficiency.
2. Row column compression through the Boolean matrix is done to reduce the scanning times of the transaction database [8,22–27]; in the process of scanning, the candidate itemset is replaced in the form of an index table, which avoids the trouble of generating a large number of candidate itemsets.
3. When searching frequent itemsets and calculating confidence, a Trie tree is used to speed up the search. A Trie tree is a data structure commonly used in data mining algorithms. This data structure occupies less memory and can quickly build and mine the effective information in the tree [28]. Many prefix tree-related technologies are applied to the algorithm of frequent itemsets mining to improve the execution efficiency of the algorithm.

### 3.2. Algorithm Procedure

Step 1. The database is traversed once and irrelevant transaction item records are deleted. The total number of transaction items is set as *m* and the traversal database as *D*. When *D*_*x*_(*x*=1,2,…, *m*)count=1, *D*_*x*_ is deleted and traversed repeatedly to get a new dataset *D*′.
Step 2. The transaction matrix is received, and the rows and columns are compressed.
The transaction dataset *D*′ is converted into matrix Mat, where transactions are sorted in column order and itemsets are sorted in row order. The matrix is represented as follows:
  (1) $$\begin{array}{c} T_{1}T_{2}\ldots T_{n},\\ \text{Mat}=\left[\begin{array}{cccc} d_{11} & d_{11} & \cdots & \;d_{1n}\\ d_{21\;} & d_{22} & \cdots & d_{2n}\\ \vdots & \vdots & \ddots & \vdots \\ d_{m1} & d_{m2} & \cdots & d_{mn} \end{array}\right]\begin{array}{c} I_{1}\\ I_{2}\\ \vdots \\ I_{m} \end{array}. \end{array}$$
If the *i*-th itemset is in the *j*-th transaction, the value *d*_*ij*_ of row *i* and column *j* of the matrix is 1; otherwise, it is 0; hence, the Boolean matrix is obtained.
Through the Boolean matrix obtained in the previous step, the support of the itemset formed by a row in the matrix can be calculated. The support is obtained by the bitwise sum operation of each row of vectors.
  (2) $$\begin{array}{c} \text{support}\_\text{count}=\;\sum_{j=1}^{n}\left(d_{i_{1}j}\cap d_{i_{2}j}\cap d_{i_{3}j}\cap \cdots \cap d_{i_{k}j}\right). \end{array}$$
According to the Boolean matrix and the calculation method of support, the support of each set is obtained, and the itemset index table is obtained. Then, the frequent itemsets are obtained by comparing them with the set minimum support.
According to the nature of frequent itemsets, if an itemset is nonfrequent, then all supersets of the itemset are also nonfrequent, which can be deleted directly, that is, row compression.
Since each transaction of the Boolean matrix corresponds to a column vector, if the length of a transaction is less than *k*, it is impossible to include *k*-frequent itemset *L_ k*. The transaction can be deleted directly during the search, that is, column compression.
Step 3. The compressed Boolean matrix is scanned again, the support is calculated, and the index table was created. The above steps are repeated until k-frequent itemsets can no longer be generated, and finally, all frequent itemsets are presented in the form of an index table.
Step 4. Finally, all frequent itemsets are searched in the form of a Trie tree to calculate the confidence, so as to generate strong association rules, that is, the association rules that users are interested in.

### 3.3. Algorithm Explanation

1. Avoid database scanning many times. The data records can be replaced with the encoded sets after only scanning the database twice. After that, all frequent itemsets can be obtained only through operations in memory. Thus, the efficiency of the algorithm is improved.
2. Binary operation is used to replace the operation between sets in the execution of the Apriori algorithm, which improves the execution efficiency of the algorithm.
3. A Trie tree is an advanced data structure that is sometimes also known as a prefix tree or digital tree. It is a tree that stores data in an ordered and efficient way. Using a Trie tree improves the algorithm efficiency.

## 4. Case Illustration

The Chinese herbal medicine data of Chinese medicine treatment for COVID-19 are selected for the experiment, and the Apriori algorithm, FP growth algorithm (FP stands for frequent pattern) and improved Apriori algorithm are compared and analyzed. The program, written in *Python* 3.8.3, simulates and analyzes the different values of other parameters of the algorithm, including support and confidence. According to the simulation results, the algorithm with strong applicability is selected and reasonable parameters are set for deeply mining the hidden association rules between Chinese herbal medicines. The simulated hardware environment is Intel (*R*) core (TM) i7-10875H CPU @2.30 GHz 16.0 GB RAM.

### 4.1. Chinese Herbal Medicine Data

This study was conducted based on the pharmaceutical prescriptions that have achieved good preventive and therapeutic effects in practice.

We searched the treatment literature on CNKI and the official treatment plan all over China. CNKI is a key national research and information publishing institution in China. Its first database was the China Academic Journals Full-text Database. In 1999, CNKI started to develop online databases. To date, CNKI has built a comprehensive China Integrated Knowledge Resources System, including journals, doctoral dissertations, masters' theses, proceedings, newspapers, yearbooks, statistical yearbooks, ebooks, patents, and standards.

The plan clearly aims at the prevention and treatment of new coronary pneumonia, until November 19, 2020, which was published on the official website of the National, Provincial, Autonomous Region, and Municipal Health Commission. The prescriptions in the plan were extracted and screened. Single Chinese medicine, incomplete composition and dosage of prescription, recommended Chinese patent medicine prescription, and prescriptions not clearly signed by the recommended prescription department or unit were excluded. Chinese medicine prevention and treatment plan are presented in Table 2. In the table, TCM means traditional Chinese medicine.

According to the National College of traditional Chinese medicine planning textbook “Chinese medicine” and the 2015 edition of “Chinese Pharmacopoeia”, the traditional Chinese medicine names entered are standardized.

### 4.2. Model Building

The Apriori algorithm, FP growth algorithm, and improved Apriori algorithm model are created, respectively. The different values of other parameters of the algorithm are simulated and analyzed, including support and confidence. According to the simulation results, the algorithm with strong applicability is selected and reasonable parameters are set to carry out the association rule mining of acupuncture treatment for COVID-19 Chinese herbal medicine data.

The modeling process includes the following: inputting sample data and modeling parameters; comparing the operation efficiency of the Apriori algorithm, FP growth algorithm, and improved Apriori algorithm under different parameter settings. According to the simulation results, the algorithm with strong applicability is selected for modeling and simulation; after processing the treatment Chinese herbal medicine database and inputting parameters, the association rules between Chinese herbal medicines are the output, and then the results of association rules are analyzed.

Using the Chinese herbal medicine dataset, the algorithm before and after optimization is simulated and compared with the FP growth algorithm, and the variation of running time with two parameters of support and confidence is analyzed, as shown in Figure 1 and Figure 2.

Figure 1 shows the comparison of the changes in the minimum support before and after the improvement. With the increase in support, the running time of the algorithm before and after the improvement is shortened. When the support is small, the running time of the improved algorithm is less than that of the Apriori algorithm before the optimization and FP growth algorithm. The greater the support, the more important the association rules are, and the shorter the running time is.

As shown in Figure 2, the comparison between the execution time of the two algorithms before and after improvement and the change of the minimum confidence parameter is shown. With the increase in confidence, there is little difference in the running time between the two algorithms. When the confidence is small, the running time of the improved algorithm is less than that of the Apriori algorithm before optimization and FP growth algorithm, and the reliability of association rules is the strongest at this time.

In conclusion, under the same database conditions and different parameter settings, it is found that the operation efficiency of the improved Apriori algorithm is significantly better than that of the FP growth algorithm, and the effectiveness of the algorithm has been fully verified. Therefore, this article applies the improved Apriori algorithm to model and simulate, and deeply mines the Chinese herbal medicine association rules. The minimum support of the parameter value is 13%, and the minimum confidence is 60%.

### 4.3. Algorithm Performance Verification and Result Analysis

According to the above operation results, 4768 association rules are obtained (such as (Shengshigao) = > (Xingren)), which represent Chinese herbal medicines Shengshigao and Xingren, the support and confidence of which simultaneous occurrence are 15% and 73%.

We extracted binary data from the original 237 Chinese herbal medicine prescriptions (Figure 3).

There were 237 Chinese herbal medicines extracted from the 242 retrieved prescriptions in the retrieved references and plans. We carried out frequency analysis, calculated the frequency of drug use in the prevention and treatment plan, and got the high-frequency core drug. The Chinese herbal medicine frequency distribution details are presented in Figure 4. Gancao, Huoxiang, Xingren, Fuling, Chenpi, Lianqiao, Maidong, Shengshigao, Jinyinhua, Huangqi, Cangzhu, Houpu, Jiegeng, Chaobaizhu, Shenghuangqi, Yiyiren, Fangfeng, Lugen, Fabanxia, and Chaihu were the top 20 frequently selected Chinese herbal medicines. As shown in Figure 4, these drugs are often used to treat colds, pneumonia, cough, and other symptoms and diseases.

### 4.4. Improved Apriori Algorithm-Based Association Rule Analysis for Itemsets of Chinese Medicine Combination Items

We investigated 4768 association rules based on the integrated Chinese medicine data. The association rules were visually presented based on the scatter plot, and the lift of a rule was the ratio of the observed support to that expected if *X* and Y were independent (Figure 5). The results demonstrated that all rules had a high lift. The association rules between different individual Chinese medicines were ordered by support. The top 20 improved Apriori algorithm-based association rules of Chinese medicine are listed in Table 3, among which, “LHS” stands for left-hand side and “RHS” stands for right-hand side. For example, No. 1 means association rule (Shengshigao)-> (Xingren) which has a support of 0.15126050, a confidence of 0.7346939, a coverage of 0.20588235, and a lift of 2.534161. This rule has occurred 36 times in the dataset.

Graph-based visualization by color or size was used for the grouped itemsets. Based on a grouped matrix of these 20 association rules, the features were visually exhibited (Figure 6). This figure clearly represented the association rules and was suitable for very small sets of rules to avoid chaotic expression.

Results showed that based on the grouped matrix evidence for 20 association rules (Figure 6), (Shengshigao) => (Xingren), (Tinglizi ) => ( Shengshigao), (Fabanxia) => ( Fuling), and (Xingren) => (Shengshigao) were interactively selected to reveal the rule's antecedent (LHS) and consequent (RHS) itemsets. By comparing with Table 3, it can be seen that the interactively selected association rules are in accordance with rule numbers 1, 2, 3, and 4.

After analysis, it is found that the highest high-frequency drugs include Gancao, Xingren, Huangqin, Lianqiao, etc. Modern pharmacology shows that glycyrrhizic acid and glycyrrhetinic acid in Gancao have antiviral effects and can significantly inhibit virus replication [26]. Modern pharmacological studies indicate that Huangqin, Lianqiao, etc. have antiviral activity, as well as cough relieving and expectorant effects. Jinyinhua is also reported to have antiviral effects [27].

Through the analysis of association rules, it is found that the medicine group with higher confidence is (Tinglizi, Xingren)-> (Shengshigao); the above medicine group plus Mahuang and Gancao can form a new group of Maxing Shigan decoction. The whole prescription has the effects of pungent cooling, lung-clearing, and asthma relieving. Among them, These are Chinese medicine treatmentterminology, such as “lung-qi,” “lowering lung” “promote qi.“ Gypsum clears and relieves lung heat, and licorice nourishes qi and neutralizes various medicines. Modern pharmacological studies have shown that Maxing Shigan decoction [27] has a wide range of effects on respiratory diseases; has good anti-inflammatory, anti-flu, and immune-improving effects; and can play the role of chemical drug oseltamivir in anti-influenza virus ceramidase activity. This prescription has been valued in the prevention and treatment of H1N1 influenza, avian influenza, and SARS, and is worthy of further clinical research and promotion.

In clinical practice, the application of traditional Chinese medicine is usually used to treat patients by using a combination of multiple traditional Chinese medicines instead of a single medicine. In the theory of Chinese medicine, for “combined” Chinese medicinal decoctions, the technical term is “compatibility,” which means to selectively combine two or more drugs, and the important thing is to determine the drug combination rather than a single drug.

## 5. Conclusion and Future Work

Aiming at the low efficiency of the Apriori algorithm, an improved association rule mining model is established in this article by mining the strong association rules between items, reducing the number of database scans, and putting forward an improved algorithm. We selected Chinese herbal medicine data for treating COVID-19 to mine hidden association rules between Chinese herbal medicines and frequent Chinese herbal medicine combinations. The simulation results showed that the improved algorithm can meet the requirements of Chinese herbal medicine association rule mining, improve the efficiency of data processing, and the reliability of Chinese herbal medicine in the treatment of COVID-19 association rule mining, and has good application value.

Besides, the algorithm used here can be further improved. The next step is to consider using the weighted Apriori algorithm if the weight is available. Furthermore, association rule analysis is just one method of data mining. Later, combining other data mining methods will be considered to reflect the association more comprehensively and objectively [29–34].

## Figures and Tables

**Figure 1:** Comparison of minimum support before and after improvement.

**Figure 2:** Comparison of minimum confidence before and after improvement.

**Figure 3:** Binary data diagram.

**Figure 4:** Distribution of Chinese medicines used in the retrieved plans.

**Figure 5:** Scatter plot for 4768 rules.

**Figure 6:** Grouped matrix for 20 association rules.

**Table 1:** Comparison of publications according to their contents.

Studies	Year	Description	Field	Characteristic of algorithm
Shumin et al. [8]	2022	Collect natural driving data, extract risk conditions, and analyze the direction and intensity of risk influencing factors with the confidence of association rules of the Apriori algorithm.	Road traffic driving	Ordinary Apriori algorithm

Weidi et al. [9]	2021	The Apriori algorithm is used to analyze the causal association rules of bridge deterioration in Yunnan Province	Bridge construction	Genetic algorithm and grey correlation analysis solve the problem of the value of support and confidence in the Apriori algorithm

Luo et al. [10]	2021	Based on the scores and employment information data of higher vocational college graduates during their school years, this article uses the Apriori algorithm to analyze the correlation between school performance and actual employment.	Education	Ordinary Apriori algorithm

Wu [11]	2019	The power optical transmission network uses the Apriori algorithm to screen and retain the alarm items and fault items that occur infrequently but are actually very dangerous.	The power optical transmission network	Weighted Apriori algorithm

Luo et al. [10]	2018	Find frequent patterns in live transportation data by using association rule mining of the FP-growth algorithm.	Public transport ride	FP-growth algorithm

Tan et al. [12]	2021	The Apriori algorithm is used to analyze the acupoint combination of acupuncture and moxibustion in the treatment of impotence	Chinese acupuncture for impotence.	Ordinary Apriori algorithm

Zhang et al. [9]	2021	The Apriori algorithm is used to analyze the acupoint combination of acupuncture and moxibustion in the treatment of optic atrophy	Chinese acupuncture for optic atrophy.	Ordinary Apriori algorithm

Lijuan et al. [13]	2016	The Apriori algorithm is used to analyze the combination of Chinese herbal medicine for treating hypertension	Traditional Chinese medicine treatment.	Ordinary Apriori algorithm

Yili Nurmaiti et al. [14]	2016	The Apriori algorithm is used to analyze the combination of Chinese herbal medicine for treating coronary heart disease.	Traditional Chinese medicine treatment.	Ordinary Apriori algorithm

Wu et al. [15]	2016	The Apriori algorithm is used to analyze the prescription containing licorice by Yan Zhenghua, a master of Chinese medicine.	Traditional Chinese medicine treatment.	Ordinary Apriori algorithm

Hai et al. [16]	2016	The Apriori algorithm is used to analyze the law of ancient laxative prescriptions.	Traditional Chinese medicine treatment.	Ordinary Apriori algorithm

Wang et al. [17]	2016	The Apriori algorithm is used to analyze the combination of Chinese herbal medicine by lidongyuan.	Traditional Chinese medicine treatment.	Ordinary Apriori algorithm

**Table 2:** Traditional Chinese medicine prevention and treatment plan.

No.	City	Plan
1	Beijing	Notice of Beijing Municipal Administration of traditional Chinese medicine on printing and distributing the “Beijing New Coronavirus Pneumonia Prevention and Treatment Program of Traditional Chinese Medicine (Trial Version 5)”
2	Tianjin	Tianjin new coronary virus pneumonia traditional Chinese medicine prevention and treatment plan (trial version 3)
3	Shandong	Notice of Shandong Provincial Health Commission on printing and distributing the “Shandong Province New Coronavirus Pneumonia Prevention and Treatment Program of Traditional Chinese Medicine”
4	Henan	Henan's new coronary pneumonia TCM prevention program
5	Gansu	Notice on issuing the prevention and control plan of traditional Chinese medicine for the normalization of the new coronary pneumonia epidemic in Gansu Province
6	Guangdong	Traditional Chinese medicine treatment program for new coronavirus pneumonia in Guangdong Province (trial version 2)
7	Shaanxi	Shaanxi issued a Chinese medicine treatment plan for pneumonia caused by new coronavirus infection (trial version 2)
8	Hunan	Rehabilitation diagnosis and treatment program of traditional Chinese medicine for patients with new coronary pneumonia in Hunan Province (trial)
	Hunan	TCM diagnosis and treatment plan for pneumonia caused by novel coronavirus infection in Hunan Province (trial version 3)
9	Sichuan	Sichuan new coronary pneumonia prevention and control guide of traditional Chinese medicine (fourth edition)
10	Jiangxi	Notice on printing and distributing the “Jiangxi Province Novel Coronavirus Pneumonia Prevention and Treatment Program of Traditional Chinese Medicine (Trial Version 3)”
11	Jilin	TCM treatment plan for pneumonia caused by novel coronavirus infection in Jilin Province (trial version 1)
12	Yunnan	Notice of the Yunnan Provincial Health Commission on printing and distributing the Chinese medicine prevention and treatment plan for pneumonia caused by new coronavirus infection (trial version 2)
13	Shanxi	Shanxi issued the “Province New Coronavirus Pneumonia Prevention and Treatment Plan with Traditional Chinese Medicine (Trial)
14	Hainan	Hainan Province new coronavirus pneumonia prevention and treatment plan with traditional Chinese medicine (public version, trial version 2)
15	Qinghai	Qinghai Province new coronavirus pneumonia prevention and treatment plan of Tibetan medicine (trial version 2)
16	Jiangsu	TCM syndrome differentiation and treatment plan for new coronavirus pneumonia in Jiangsu Province (trial version 3)
17	Ningxia	Ningxia Hui autonomous region new coronavirus pneumonia prevention and treatment plan with traditional Chinese medicine (trial)
18	Hebei	Notice on printing and distributing the pneumonia diagnosis and treatment plan for new coronavirus infection in Hebei Province (trial version 2)
19	Heilongjiang	Heilongjiang Province new coronavirus pneumonia prevention and treatment plan with traditional Chinese medicine (second edition)
20	Zhejiang	Zhejiang Province new coronavirus pneumonia recommended Chinese medicine prevention and treatment plan (trial version 4)
21	Guizhou	Guizhou Province new coronavirus pneumonia prevention and treatment of traditional Chinese medicine reference plan (second edition)
22	Chongqing	Recommended plan for the prevention and treatment of new coronavirus pneumonia in Chongqing with traditional Chinese medicine (trial version 2)
23	Mongolia	Notice of the office of the Inner Mongolia autonomous region Health Commission on printing and distributing the inner Mongolia autonomous region new coronavirus pneumonia Chinese medicine diagnosis and treatment plan (trial version 2)

**Table 3:** Top 20 Improved Apriori algorithm-based association rules of Chinese medicines.

No.	LHS	RHS	Support	Confidence	Coverage	Lift	Count
[1]	(Shengshigao)	-> (Xingren)	0.15126050	0.7346939	0.20588235	2.534161	36
[2]	(Tinglizi) ->	(Shengshigao)	0.10504202	0.8620690	0.12184874	4.187192	25
[3]	(Fabanxia)	-> (Fuling)	0.10504202	0.7352941	0.14285714	2.573529	25
[4]	(Tinglizi)	-> (Xingren)	0.09663866	0.7931034	0.12184874	2.735632	23
[5]	(Chishao)	-> (Gancao)	0.09243697	0.8461538	0.10924370	2.165426	22
[6]	(Shengdihuang)	->(Shengshigao)	0.09243697	0.7857143	0.11764706	3.816327	22
[7]	(Caoguo)	-> (Cangzhu)	0.08823529	0.7000000	0.12605042	3.702222	21
[8]	(Shengdihuang)	-> (Gancao)	0.08403361	0.7142857	0.11764706	1.827957	20
[9]	(Shengshigao, Tinglizi)	-> (Xingren)	0.08403361	0.8000000	0.10504202	2.759420	20
[10]	(Tinglizi, Xingren)	->(Shengshigao)	0.08403361	0.8695652	0.09663866	4.223602	20
[11]	(Mahuang)	-> (Xingren)	0.07983193	0.8636364	0.09243697	2.978920	19
[12]	(Fuling, Xingren)	-> (Huoxiang)	0.07983193	0.7600000	0.10504202	2.318974	19
[13]	(Huoxiang, Xingren)	-> (Fuling)	0.07983193	0.7600000	0.10504202	2.660000	19
[14]	(Wuweizi)	-> (Maidong)	0.07563025	0.7826087	0.09663866	3.801242	18
[15]	(Bohe)	-> (Lianqiao)	0.07563025	0.7826087	0.09663866	3.267735	18
[16]	(Binglang)	-> (Caoguo)	0.07142857	0.9444444	0.07563025	4.492593	17
[17]	(Baizhu)	-> (Chenpi)	0.06722689	0.8000000	0.08403361	3.022222	16
[18]	(Chenpi, Dangshen)	-> (Fuling)	0.06722689	0.8888889	0.07563025	3.111111	16
[19]	(Dangshen, Fuling)	-> (Chenpi)	0.06722689	0.8000000	0.08403361	3.022222	16
[20]	(Fuling, Houpu)	-> (Huoxiang)	0.06722689	0.7619048	0.08823529	2.324786	16

## Data Availability

The authors confirm that the data supporting the findings of this study are available within the article.

## References

[1] Su Y. (207). Internal value and development ideas of traditional Chinese medicine. *Journal of Zhejiang University of Traditional Chinese Medicine*.

[2] World Health Organization (2020). WHO Director General’s Remarks at the media Briefing on 2019-nCov on 11 February 2020[EB/OL. https://www.who.Int/dg/speeches.

[3] Zhou F., Cai W., Li X., Zhang D., Zhou Y., Zhang C. (2020). to explore the TCM Prevention and treatment strategy of covid-19 from the perspective of publicity, clearing, harmony and transformation. *Journal of traditional Chinese Medicine*.

[4] Shi S., Zhang X., Wang B. (2021). research progress of TCM intervention on sequela of new coronavirus pneumonia in convalescence stage. *Journal of Nanjing University of traditional Chinese Medicine*.

[5] Zang M., Ren J., Zhang Y. (2020). Research Progress on prevention and treatment of New Coronavirus pneumonia by Chinese and Western medicine. *World science and technology - modernization of traditional Chinese Medicine*.

[6] Liu R., Huang Y., Luo J., Xie S., Xie C, Tang J. (2021). application of Chinese medicine in the prevention of new coronavirus pneumonia (COVID-19). *Medical diet and health*.

[7] Roberto J., Bayardo R. A. Mining the most interesting rules.

[8] Shumin F., Luo M. (2021). Analysis of employment situation of higher vocational college graduates based on Apriori algorithm. *China Arab Technology Forum*.

[9] Weidi E., Zhang B., Qi X., Chen G. (2021). Acupoint regularity of acupuncture and moxibustion in treating optic atrophy based on. *R language*.

[10] Luo M., Demir-Alan U., Birant D. (2018). Server-based intelligent public transportation System with NFC. *IEEE Intelligent Transportation Systems Magazine*.

[11] Wu Y., Peng W., Huang S. Fault diagnosis of power optical transmission network based on weighted Apriori algorithm.

[12] Tan Z. G., Zhong F., Wen-ying S. H. I. (2021). Analysis on the Acupoint Prescriptions for Impotence Treated with Ancient Acupuncture and Moxibustion Treatment Based on Data Mining Technology. *Chinese Acupuncture and Moxibustion*.

[13] Zhu L., Li Y., Zhang S., Jiang F. (2016). Analysis of the medication law of hypertension prescriptions based on data mining. *Modern Distance Education of Chinese Traditional Medicine*.

[14] Yili-nurmaiti M., talipu A., mijiti E., turhong A. S. I. M., Abduriem A. (2016). Discussion on the prescription formation law of coronary heart disease prescriptions based on data mining. *Chinese Journal of Traditional Chinese Medicine*.

[15] Wu J., Guo W., Zhang X., Zhou W., Zhang Y., Zhang B. (2016). Based on data mining, Yan Zhenghua, a master of Chinese medicine, studied the prescription medication law containing licorice. *Chinese Journal of Traditional Chinese Medicine*.

[16] Lan H., Chen F., Yu X., Bian W., Zhan Q. (2016). Zhao Guoping Analysis of the medication law of ancient laxative prescriptions based on data mining. *Beijing Traditional Chinese medicine*.

[17] Wang Y., Lv J., Tian X., Li D. (2016). Research on the medication law of lidongyuan based on data mining. *Chinese Journal of Traditional Chinese Medicine Information*.

[18] Pang-Ning T., Michael S., Vipin K. (2011). *Introduction to Data Mining*.

[19] Nie P., Li Y., Wang Y., Zhang H., Guo J. (2021). Extraction method of reservoir optimal operation rules based on Apriori algorithm. *Water conservancy and Hydropower Technology (Chinese and English)*.

[20] Liu F., Wu G. (2018). an improved Apriori algorithm based on compressed matrix. *Journal of Shandong University (Engineering Edition)*.

[21] Feng S., Wu Di, Sun Y. (2021). Cause analysis of typical risk scenarios based on natural driving data. *Journal of Chongqing Jiaotong University (NATURAL SCIENCE EDITION*.

[22] Hu W., Wang W., He X., Zhang H. (2021). Multi objective causal analysis method for bridge deterioration. *Computer and digital engineering*.

[23] Ning X., Guo H., Ma R., Miao M., Zhu P. (2022). Study on medication characteristics of traditional Chinese medicine in the treatment of peptic ulcer based on data mining. *Chinese herbal medicine*.

[24] Gong hengpei, Yu E., Zhu L., Mei Y., Xu F. (2022). Analysis on the medication law of traditional Chinese medicine in the treatment of leukemia based on data mining. *New traditional Chinese medicine*.

[25] Wu A., Liu A. (2019). improvement of Apriori algorithm based on boolean matrix reduction. *Computer engineering and science*.

[26] Wang M., Rui F. (2018). Zou Shurong Improved Apriori algorithm based on matrix multiplication. *Computer and digital engineering*.

[27] Li W. (2017). Zhu Zhaoyuan an Apriori algorithm based on parallel matrix with clear target. *Journal of Zhejiang University of technology*.

[28] Zhou K., Gu H., Li A. (2018). Improved algorithm of Apriori algorithm based on association rule mining. *Journal of Shaanxi University of Technology (NATURAL SCIENCE EDITION)*.

[29] long Li, Liu P., Zhang K. (2019). Research and application of improved Apriori algorithm. *Computer and digital engineering*.

[30] Qu R., Zhang T. (2017). Improved Apriori algorithm based on matrix compression. *Computer engineering and design*.

[31] Miao M., Wang Y. (2013). Research on the improvement of Apriori algorithm based on matrix compression. *Computer engineering and application*.

[32] Bodon F. Surprising results of trie-based FIM algorithms.

[33] Yang L., Gao H., Zhu Q. (2017). Research progress on antiviral activity of licorice chemical components. *Shandong Journal of Traditional Chinese Medicine*.

[34] Liu C. (2020). The effect of Maxing Shigan Decoction in the clinical treatment of children with bronchial pneumonia and its influence on inflammatory indexes. *Psychological Monthly*.

